# Deep Neural Network Model Construction for Digital Human Resource Management with Human-Job Matching

**DOI:** 10.1155/2022/1418020

**Published:** 2022-05-19

**Authors:** Qing Ni

**Affiliations:** School of Business, Anhui University, Anhui, Hefei 230601, China

## Abstract

This article uses deep neural network technology and combines digital HRM knowledge to research human-job matching systematically. Through intelligent digital means such as 5G communication, cloud computing, big data, neural network, and user portrait, this article proposes the design of the corresponding digital transformation strategy of HRM. This article further puts forward the guaranteed measures in enhancing HRM thinking and establishing HRM culture to ensure the smooth implementation of the digital transformation strategy of the HRM. This system uses charts for data visualization and flask framework for background construction, and the data is stored through CSV files, My SQL, and configuration files. The system is based on a deep learning algorithm for job applicant matching, intelligent recommendation of jobs for job seekers, and more real help for job applicants to apply for jobs. The job intelligent recommendation algorithm partly adopts bidirectional long and short-term memory neural network (Bi-LSTM) and the word-level human post-matching neural network APJFNN built by the attention mechanism. By embedding the text representation of job demand information into the representation vector of public space, a joint embedded convolutional neural network (JE-CNN) for post matching analysis is designed and implemented. The quantitative analysis method analyzes the degree of matching with the job.

## 1. Introduction

New digital technologies such as 5G communication, artificial intelligence, blockchain, cloud computing, and big data are rapidly spreading and exploding worldwide. In this case, the “user” (not only people but also machines) continues to generate massive amounts of data, and the amount of data generated by devices is also increasing [1]. Data are generated and shared when “smart” home appliances communicate with their home servers. Examples of this include data generated by geolocation services, Web browser history, social media activity, and even fitness apps. Industrial machinery in factories worldwide is increasingly equipped with sensors that collect and transmit data, forming the Internet of Things to generate data [2]. Today, anything we do online, be it interacting with friends on social media or using a smartphone, create data on personal use and almost always leaves a digital marker. Information technology has also developed rapidly in recent years, and technology is improving [3]. Top-level designs have been released to provide the basis for the development of big data technology, marking a period of rapid expansion in the development of applications within big data. With the times, enterprises also improve their management and business through advanced digital technology.

Under the background of the new era, talents are becoming more and more strategic resources to promote economic and social development, and skills are gradually surpassing capital to become the scarcest resource in the current society and its core position in the process of enterprise development with increasing value [4]. With the deepening of modern management research, enterprise human resource management has become one of the most critical modules in contemporary enterprise management. A scientific and complete human resource management system is a crucial prerequisite for the sustainable development of enterprises [5]. Matching human resources with jobs is of great significance to the sustainable and healthy development of human resources management and modern enterprises. On the other hand, recurrent neural networks are good at modeling long sequences of text. The addition of gate control dramatically enhances the contextual power of recurrent neural networks and is widely used in semantic annotation, machine translation, and other fields. The core of man post matching is to put the right person into the proper position through suitable selection, training, assessment, motivation, and other methods so that the people and places of the whole enterprise are highly matched and operate efficiently to maximize the value of the employees and maximize the productivity of the positions. This highly checked state needs to be constantly adjusted and maintained through accurate prediction to make people and places consistent [6]. At the same time, it also enables enterprises to maximize employees' motivation and improve the whole enterprise's operational efficiency.

In recent years, most companies have embarked on digital HR management. The HR digital platform has become an essential item in the training courses for the employees of the companies. With the support of digital technology, enterprises can take the initiative to break the industry barriers and carry out multidimensional strategic policy layouts by making human resource management a specialized task and establishing a perfect and independent database with a large amount of data as the foundation. Large- and medium-sized enterprises have used digital technology to integrate and standardize their operational processes and form a complete set of digital methods, which is undoubtedly a valuable experience in developing and applying digital technology [7]. This means that there are already more and more enterprises whose HR management digitalization is gradually returning to rationality and maturity and is entering the stage of deep and meticulous cultivation. Digital technology can help companies provide the underlying technical support in talent value management so that business managers and HR departments can focus more on people. In short, companies should actively consider how they can use digital initiatives to help transform their HR management to work together to serve their strategic goals.

## 2. Related Works

As the recruitment market becomes more diverse and presents many opportunities and challenges for talent attraction, Farm examines the correlation between multiple sources of talent acquisition today and the cost, quality, and time to hire, demonstrating that the efficient use of multichannel recruiting methods is essential for the success of candidates and companies [8]. With the accumulation of online data in the talent attraction segment, researchers have focused on recruitment market trend analysis to help companies develop macro talent acquisition strategies. For example, Deepak et al. extracted skill themes from the job requirement texts by crawling the readers of recruitment requirements posted by different companies on job boards and using probabilistic topic modeling [9]. Then a serialized implicit factor model was designed to predict the future trend of other companies' demand for different skill-demanding jobs by modeling the evolution pattern of skill themes in different companies under different types of jobs. Campbell et al. wanted to model the recruitment competition problem existing in other companies for different jobs [10]. The authors use the career chain data of employees in Linkedln data and then calculate the talent flow matrix between companies and positions under different periods to represent the competition phenomenon existing in the recruitment market at different periods and design a model based on tensor decomposition to predict the competition trend in the future market, i.e., the talent flow matrix at future moments, to help companies find the most urgent talents at present. This will allow companies to find the most critical skills and develop talent attraction plans in a targeted manner.

The person-job matching direction also has many researchers doing related research. Troth and Guest et al. compared some user-based collaborative filtering and project-based collaborative filtering algorithms for a job recommendation. Recently, various online recruitment services have provided a new perspective for recruitment analysis [11]. For example, Trullen et al. proposed the generalized linear mixed model (GLMix) in the LinkedIn job recommendation system, a more fine-grained model at the user or project level, resulting in 20% to 40% more job applications generated in the system [12]. Yabanci collected job-related information on various social media to construct inter-company job-hopping network relationships and demonstrate talent mobility [13]. Pak et al. used employee career path data to predict employee job changes [14]. Zeebaree et al. proposed a talent circle discovery model based on job change networks to help companies find the right talent and provide career advice to job seekers to find the right job [15]. Collins used BP neural network theory to establish a human-job matching assessment model and conduct simulations to verify BP neural networks' robust self-organization, self-adaptation, and self-learning capabilities to evaluate the human-job matching situation technology personnel scientifically and effectively in enterprises [16]. Steffensen et al. proposed a precise matching algorithm combining deep semantic features. Constructing a complete human-job feature system, they used natural language processing technology and the Doc2vec method to fully explore the semantic information in long texts to achieve precise matching between job seekers and jobs [17].

Current representative research in the digitalization of HRM focuses on several areas: some focus on the development and design of HR systems. Digital technology can influence the way business is governed and even change the shape of the company, such as transaction processing, decision-making, and office work. Various industries have begun to implement digital management, such as the feasibility of establishing a human resource management information system for coal mining enterprises and issues related to its development and application, as well as proposing a framework for a university management information system based on the ASP system; structural theory, which views digital technology as a supporting structural feature, asserts that it may be difficult to accurately capture the relationship between technology and people in the current context. Some scholars aim to explore to improve their value in the information age [18]. Enterprises should adjust from human resources, break the traditional management model and management concept, and use scientific management methods and computer network technology to realize information and digital human resource management. Chen Yao believes that the use of information should be used throughout the process of personnel management and decision-making, and Liang Han et al. believe that HR management information system is a critical way to promote organizational development. Other scholars believe that constructing HRMIS can efficiently manage and retain talents and discuss how HRMIS plays a role in managing and controlling skills.

## 3. Designing a Deep Neural Network Model for Digital Human Resource Management to Match People and Jobs

### 3.1. Digital Human Resource Management System Design

Human resource management is the traditional pyramid model; this model divides human resource management by function. The work of each functional module is divided into three parts: essential transactional work, HR practical module work, and strategic change work. The advantage of this model is that the division of responsibilities of each position is clear, and the result is easier to carry out. Each module becomes an isolated individual, and there is little connection between them, leading to the company's HR spending most of its energy on administrative work. It is not easy to provide strategic support to the organization. Therefore, most of the time, the company's HR department is treated as an administrative service department. It is believed that they only increase the cost but do not create profit, and the business demand in this model is not very big, and it can only meet the needs of the company in the initial growth stage. As the organizational scale of the company continues to expand, when the business departments put forward their demands, each HR function of the company provides solutions or implements policies on the modules they are responsible for. This rigid division either fails to reach the overall direction of the business departments or lacks flexibility and maneuverability. Therefore, the traditional operation mode of dividing teams by function (such as compensation, training, and performance) can no longer keep up with the company's current development needs. According to the new “three-pillar” management model with the shared service center as the grip, the company's HR department operates as a business department. The customers it serves are the internal business departments. At the same time, the needs of customers are finely divided. Through the “three pillars” management model, the three roles support each other and work closely together to better play their supporting roles in business and strategy, generate more added value, and make more significant contributions to the company. The HRM function diagram is shown in Figure 1. As the organizational scale of the company continues to expand, when the business departments put forward their demands, each HR function of the company provides solutions or promotes policies on the modules they are responsible for. This rigid division either fails to meet the overall needs of the business departments or lacks flexibility and mobility.

HR teams' ineffective use of analytics tools is primarily limited by data collection. With the support of today's data analytics software, which supports a variety of data from different data sources, thus avoiding the need to change source systems or perform large-scale data modeling and integration. HR departments can integrate business and HR data, use technology to create relevant assessment metrics, monitor HR productivity and its impact on the business, and thus gain insight into employee capabilities and needs, and optimize HR management processes. Digital technology can help companies provide the underlying technology support for talent value management so that business managers and HR departments can be more people-focused. We use quantitative analysis as a critical entry point to transform the company's digital HR and show the status of implementing the three-pillar HR management model in real-time to provide adequate support for decision-makers in designing and optimizing solutions. The HR team can improve the match between talent strategy and business needs through a more forward-looking management approach by grasping the company's historical trends [19]. Positive feedback refers to the interaction between objects, creating a joint propulsive force that will strengthen the original development trend, and create irreversible inevitability. By setting up quantitative indicators on the company's implemented HR SSC and adopting quantitative analysis methods with the help of data and system integration, the company's managers can gain insight into the status of the company's HR management. It is necessary to establish a positive feedback mechanism, HR SSC generates data, and the integrated data reverse to promote HR SSC optimization and improvement. The SCC system job data set is shown in Figure 2.

The project team developed the following design content based on business orientation, quantitative analysis, and positive feedback. Based on the current human resource situation of the company and the future development direction of the company's business, the transformation direction of human resource management was clearly defined as shifting from the traditional hybrid to the three-pillar model. By analyzing the correspondence between the three pillars and each functional module, the relevant work of each module is embedded in each pillar of the three-pillar model to ensure that each pillar has work related to the functional module, such as recruitment, training and development, performance management, compensation, and benefits. The focus of each pillar in the human resources function is different. By analyzing the quantitative indexes of the four aspects of human resource management of the company, namely “selection, training, employment, and retention,” we deepen our understanding of the status of human resource management and then take targeted measures to optimize and improve the weak links, enhance the operational efficiency of human resource management, improve the level and quality of service of the HR department of the company, and contribute to the achievement of the company's business goals. The basic reports and analysis indicators of HR are sorted out to form a common enterprise analysis system [20]. The feedback mechanism of “positive promotion” takes the business target of Company F as the first choice, subdivides the target into performance indicators, sets up performance indicator targets through industry benchmark values and historical values of the company, and distributes the performance indicator targets to departments and responsible persons. Regularly summarize the actual situation of performance indicators, understand the current operation level of each business organization, compare the difference with the target, and corporate executives communicate comprehensively from financial, human structure, company atmosphere, and leadership aspects, find solutions through internal and external communication and sharing, and improve human resource management through continuous optimization and improvement of performance. The best management ideas must be landed through the HR system. The extensive database related to corporate human resources is generated based on data specification and process specification to make the digital management of human capital landed. In the application process of the company system, the index data from the group to each branch should be standardized to ensure the accuracy of the results. HRM operations are divided according to the three roles in the three-pillar model. Since theoretically, the three role functions are divided into clear boundaries, but in the actual process, it is impossible to divide them clearly, and they cannot be separated during business execution, the HR operations management function is established explicitly for information integration and operations management, and divided into HR SSC. At the same time, a part of employee relations and personnel handling, which is theoretically a COE function, is put under HR SSC. Thus, HR SSC takes over the three functions and provides strategic guidance for establishing the future system. The specific role of division and operation management functions are shown in Figure 3. The core of man post matching is to put the right person into the correct position through suitable selection, training, assessment, motivation, and other methods so that the people and places of the whole enterprise are highly matched and operate efficiently to maximize the value of the employees and maximize the productivity of the positions. This highly checked state needs to be constantly adjusted and continuously maintained through accurate prediction to keep the best configuration of people and places. At the same time, it also enables the enterprise to maximize the employees' motivation and improve the whole enterprise's operational efficiency.

### 3.2. Human Post-Matching Deep Neural Network Model Construction

The matching problem of job requirement information is ultimately a text mining problem. Since tags have two features, semanticization and short text, and job requirement information is also relatively standardized and formatted text information, the human-job matching problem in this article can be classified as a natural language processing (NLP) problem. Traditional text mining methods require a lot of manual characterization engineering and feature selection work, and this labor-intensive approach is backward in the context of big data. With the continuous development of deep learning, convolutional neural networks (CNNs) and recurrent neural networks (RNNs) point to new directions for text mining. A dynamic convolutional neural network model for sentence representation has been proposed and achieved surprising results on many text classification problems. The power of CNNs for natural language processing using only one convolutional layer has been demonstrated.

On the other hand, recurrent neural networks are good at modeling long text sequences. The addition of gate control dramatically enhances the context control of recurrent neural networks and is widely used in semantic annotation, machine translation, and other fields. The job requirement information data characteristics of this article are labeled, hierarchical, and discrete [21]. The data primarily consists of short sentences or limited keywords, and the dependence on serialization is not apparent. The CNN model can mainly discover the hierarchical and local semantic features of the text. At the same time, the RNN is primarily good at finding the sequential features and global features of the text. Therefore, this article considers that convolutional neural networks are more suitable for solving human post-matching analysis problems than recurrent neural networks. The text CNN mainly has four layer structures such as input layer, convolutional layer, pooling layer, and fully connected layer. The design of the convolutional neural network model is shown in Figure 4. HRM is a traditional pyramid model, this model divides HRM by function, and the work of each functional module is divided into three parts, which are essential transactional work, HR practical module work, and strategic change work.

Input layer: the input consists of a set of document matrices of size *N* × *K*, where *N* represents the number of words in the document and *K* denotes the dimensionality of the word vector. Convolutional layer: the convolutional layer mainly performs convolutional operations and consists of convolutional kernels of different sizes. The dimension of the convolution kernels is *m* × *K*, where *m* denotes the height of the convolution kernels. The document matrix is convolved with the size of the convolution kernel as a sliding window. There are as many feature vectors as convolution kernels; each can discover one feature in one kind of text matrix. Pooling layer: the pooling layer is a downsampling of the output of the convolutional layer, which can unify the dimensionality of text sentences of different lengths. The two main pooling methods are average pooling (taking the average of each vector feature) and maximum pooling (taking the most value of each vector feature). The pooling operation allows discarding unimportant positional feature information while retaining the local information captured by convolution. Fully connected layer: the pooling output is weighted and passed through a softmax classifier to obtain the probability of classifying a document into each category, thus the final classification result. This layer usually incorporates a dropout mechanism, where each connection is discarded with a small probability, enhancing the model's generalization ability. The objective of a standard text convolutional neural network is a cross-entropy function with the following equation.

(1) $$\begin{array}{c} l=\sum \left(x-y\right)\text{log}\left(\frac{x-y}{P}\right),\\ \text{log}\left(\frac{x-y}{P}\right)=\text{log}\left(\sum_{K}\frac{j-1}{\exp\left(y_{i}\right)}\right). \end{array}$$

There are two main uses of text convolutional neural networks in this article. One is text modeling of short texts in student portrait labels and job requirement information, i.e., the construction of word vectors. Since the wording of job requirement information is relatively concise and the descriptions of similar job requirements are the same, the richness of the portrait labels in this article is higher than that of job requirement information. The second is to realize the human-job matching analysis. This article will propose an objective function that meets the characteristics of this article and use a more effective optimization method to complete the training of the joint embedded convolutional neural network (JE-CNN). Calculating the similarity of human post-matching cases requires ontology semantic similarity calculation based on concept names to filter out the initial set of available instances [22]. The similarity of concept names includes the likeness of ontology and attribute names, where the ontology names are used to determine whether the ontologies in different cases describe the same class of things and objects, for example, whether they both represent the development engineer class or the 5G development engineer position. Attribute names determine whether the attributes' names match when two ontologies describe the same type of things and objects. We use quantitative analysis as a critical entry point for transforming the company's digital human resources and showing the status of the “three-pillar” HR management model in the company in real-time to provide adequate support for decision-makers to design and optimize solutions.

(2) $$\begin{array}{c} \text{Sim}\left(\frac{o_{1}A}{o_{2}A}\right)=\frac{\sqrt{o_{1}-o_{2}}}{o_{1}+o_{2}}. \end{array}$$

The calculation of concept name similarity can narrow the scope of case retrieval, reduce the space of case retrieval, and get a rough alternative case set based on the calculation results. Still, each concept has many characteristic attributes, and the number of attribute values is much larger than the number of images. To filter cases based on the distinct attribute values of patients, it is also necessary to calculate the attribute similarity between cases. In the CBR case retrieval layer, after the initial screening case set of human post matching is obtained through ontology concept retrieval, the attribute-based similarity calculation between the target cases and the source cases in the initial screening case set is needed to realize the case retrieval and matching. The attribute features of CPPF mainly refer to the problem description (P Analysis), situation description (R Analysis), etc., of the case. In CPPF records, there are two forms of attribute similarity calculation, attribute text feature type, which is used to express the attribute features of cases that are difficult to be described by numbers or vocabulary; attribute value type includes exact value type, that is, the actual number accurately expresses the attribute characteristics of the case, and interval type is the concept of specific interval value, which is often used to describe the attribute characteristics of the case. The similarity of the attributes of the matter is denoted as the similarity of the textual characteristics of the case. The similarity of attribute text features is recorded as attribute text, which is mainly a combination of feature extraction based on the TF-IDF algorithm and dimensionality reduction based on LDA topic model training to calculate the similarity between two different job matching cases when an attribute value is a text, i.e., the proportion of the number of extracted standard text features to the number of all text features, in the job matching cases, the attribute text features. Digital technology can help companies provide the underlying technology support for talent value management so that business managers and HR departments can be more people-focused.

(3) $$\begin{array}{c} {\text{Sim}}_{at}=\sqrt{\frac{N\left(P_{0}\right)-1}{N\left(P_{0}\right)+N\left(P_{i}\right)}}. \end{array}$$

Here *N*(*P*_0_) denotes the set of text features extracted from attribute *P* in the target case, the attribute text feature similarity is determined by the ratio of the number of standard text features of the same attribute in the set of all text features in the two cases. The greater the value of the common feature attributes shared by two instances in the same point, the higher the similarity. The precise numerical similarity mainly calculates the accurate numerical value in job attribute features of the man-job matching cases. Exact numerical values represent the attribute features of the concept nodes. After the search based on the concept name, the points in the initial screening of the case set are further calculated for the precise numerical similarity. The attributes are quantitatively determined, and their numerical attribute similarity is: by making human resource management a specialized task while establishing a sound, independent database and having a large amount of data as a foundation, supported by digital technology, companies can take the initiative to break industry barriers and layout a multidimensional strategic approach.

(4) $$\begin{array}{c} {\text{Sim}}_{av1}=\sum \left(\frac{\sqrt{x-y}}{\text{Max}\left(x\right)-\text{Min}\left(y\right)}\right)+1. \end{array}$$

Max-Min denotes the interval range of the values taken by the human-job matching caste features, and *x* and *y* represent the specific values of a feature attribute in the CPPF _0_and CPPF_*i*_, CPPF_*i*_ of the human-job matching case. Since different job attribute features and case attribute information have other effects on the retrieval results in the similarity calculation, weights need to be introduced and combined with the weight assignment opinions of the domain to ensure the objectivity and accuracy of the job feature identification results experts. The weighted attribute similarity is obtained by attribute text feature similarity calculation and attribute numerical similarity calculation, expressed as most enterprises have embarked on the construction of HR digital management. The HR digital platform has become an essential item in the training courses for the enterprises' employees and is fully used in the actual work.

(5) $$\begin{array}{c} {\text{Sim}}_{\text{add}}=\sum_{1}^{i}wi-w_{i}, \end{array}$$

where *w*_*i*_ denotes the weight of each different attribute and ∑_1_^*i*^*wi*, according to the attribute similarity calculation, the similar case set CPPF is extracted ^A^from the preliminary available source case set CPPF^R^. After the case retrieval is completed, the matching case set may not precisely match the target case. The source case needs to be modified and updated to make it more compatible with the requirements of human-job matching.

## 4. Analysis of Results

### 4.1. Analysis of the Digital Human Resource Management System

The HR information system will play a vital role in the HR digital management construction process. Even a good management idea must be landed through the HR system. An extensive database related to corporate human resources is generated based on data specification and process specification to make the digital management of human capital landed. During the application of the company system, the index data from the group to each branch should be standardized to ensure the accuracy of the results. The company should unify the unit organization, position, employment determination, compensation, and welfare management. Establish a value creation-oriented, reasonable structure, and standard compensation system and consolidate the achievements of compensation reform. In addition, the company should also unify the employment management system, use information technology to implement human resource planning, fulfill the responsibility of human resource development and allocation, and implement the organization, staff, performance, and salary management system strictly and effectively. The salary range of Internet IT positions is shown in Figure 5.

By optimizing each functional module, the department's workforce needs can be quickly analyzed, and the quality and functionality of digital technology can be fully utilized in the development of human resource management practices. Human resource planning is a compelling content and component of the company's human resource management and essential infrastructure and supports ineffective action. In human resource planning, the company mainly analyzes the supply and demand of employees and human resource management needs [23]. In the context of the information age, the tedious staff planning process of the past can be changed by implementing digital control in the actual execution of planning work. The cloud-based resources of big data can implement effective integration and workforce allocation in the marketplace. It enables the existing HR digital management platform to align with the development strategy. It can finally meet the daily required operation habits and business processes to become a qualified, advanced, and efficient management platform. The job data map is shown in Figure 6.

Comprehensive analysis of the existing job system structure and job characteristics, and fully considering the company's actual development needs, targeted human resources management strategy to improve the efficiency of enterprise human resources management. Enterprise straightforward job-post system structure would be more conducive to clear employee qualifications, performance standards, apparent job difficulties of each position, and effectively avoids the situation of employees shifting responsibilities to each other. According to the development strategy of Company A, a promising talent supply chain is established, which allows the company to save a lot of time and money in human resource planning and management so that the specification and management of human resources are consistent with the actual demand. It provides a better logistic guarantee for top-level decision-makers, middle-level management, and staff development. It can be essentially close to its digital development strategy of human resources. The trend graph of the number of employees is shown in Figure 7.

### 4.2. Human Post-Matching Deep Neural Network Model Construction Implementation

The ontology-based person-job matching case reasoning system is a kind of knowledge intelligent reasoning system to solve the problems of knowledge service, job and personnel matching prediction, and job competency feature identification in the process of person-job matching work in the field of human resource management. To verify and realize the research results in the previous chapters of this article and also to provide methods and technical support for improving the rational allocation of enterprise knowledge-based employees and positions, this article designs and implements a human-job matching case reasoning system based on the ontology of job competency characteristics, and the functions provided by this matching system are: knowledge service for human-job matching of enterprise knowledge-based employees, knowledge management of human-job matching, and competency matching of job requirements. The matching system provides the following functions: knowledge service of job matching for enterprise knowledge-based employees, knowledge management of job matching, prediction of competency matching of job requirements and personnel, automatic identification of competency characteristics of job requirements, and precise matching of human and job positions. The automatic identification and matching of competency characteristics of job requirements for knowledge-based employees is the most crucial part of the development process of the man post-matching system. The module extracts the most vital information from job name, job level, job nature, salary range, job content, job category/type, nature of the enterprise, enterprise-scale, industry category, location, and other aspects according to the knowledge module and the competency model of job competency characteristics, combined with the setting of similarity threshold. The features of the most similar cases are extracted from the situation of job title, job level, job nature, salary range, job content, job class/type, nature of the enterprise, enterprise-scale, industry category, region of the enterprise, etc., and used for the automatic identification of the competency features of enterprise knowledge employees' job requirements based on ontology and case inference, to get the human-job matching solution quickly and accurately. The label prediction results are shown in Figure 8.

To verify the feasibility and effectiveness of an artificial job matching case-based intelligent reasoning system, the system is tested through a specific retrieval example of an artificial job matching problem. Log in to the account by username and password, enter the manual job matching case-based reasoning system, summarize the relevant information of the target case, and input the attribute characteristic form of the adult job matching case. According to the indicators and their weights provided by the user profile, the user first evaluates the explicit knowledge of the candidates, sets thresholds, and selects some candidates for matching. Then the system requires users to input the content about evaluating candidates' tacit knowledge (to be developed), and the comprehensive evaluation of candidates is generated by combining tacit knowledge measure and similarity ranking with users' personal data, and the job matching, case-based reasoning, and candidate screening are completed. For different categories of jobs, the model performs differently. For technical positions, the AUC performance of this model is relatively good, while for other types and civil service, the performance is relatively weak. The main reason is that the technical category focuses more on the accumulation of students' specialized behaviors in school, and the professional skills requirements are relatively straightforward, which can be better reflected in the portrait. There are generally no precise skill requirements for public service and other categories. Some even apply for jobs through additional exams, such as civil servants in government departments, which require rigorous exams on the one hand, and a meager recruitment ratio on the other. Therefore, the relevance of these two types of jobs to the portrait is low. With the deepening of modern management research, enterprise human resource management has become one of the most critical modules in contemporary enterprise management. A scientific and complete human resource management system is a crucial prerequisite for the sustainable development of enterprises. To better reflect the model's value, the guiding role of man post matching the job part is relatively sparse. More independent between different requirement items, job demand information is usually published to the public after careful examination. The wording is fixed single, leading to a remarkable similarity between different companies describing similar jobs. Still, the requirements of other companies are additional. In this article, the company name is also used as input. The items can be adjusted on the vector merge to distinguish the similar requirements of different companies. The effect under the additional data cut ratio is shown in Figure 9.

In terms of dimensions, items 2,4,6,7 are relatively sparse and small. On the one hand, “ability to apply cutting-edge artificial technology and algorithms,” “spirit of challenging impossible and innovative,” and “good at communication” appear in most of the job requirements are considered essential requirements. On the other hand, the value of the dimension “TensorFlow, Caffe, MATLAB” is relatively small and sparse because of the rapid changes in the Internet and artificial intelligence, the degree of modification of various framework technologies is relatively large, and students who master different framework technologies for the same type of positions can be matched smoothly. Hence, the value of this dimension is small and sparse, and the framework of similar roles, such as web-related positions, is rich and fast-changing. It should be noted that since the subjective labels are textualized, so each personal title is identical, their emotional label vector will be the same. Therefore, this article regards these as the baseline vector, while the behavioral label vector can be the bias vector. However, the network's input is richer than that of the graph; for example, “profession,” “gender,” etc., are also used as input, then the baseline vectors will become more diverse. For the matching analysis, the cosine similarity of the overall vectors is 0.7818 calculated, and the resemblance is increased to 0.8131 if the behavioral labels are partially removed. In the AUC calculation of the general sample, to choose a better classification threshold, it is necessary to use an index. This Jorden index is determined in this article using MATLAB's ROC function. The classification threshold is 0.5819 decided as to when the cosine similarity of the person and the job is more significant than this value; the model considers that the two can match successfully, while less than this value indicates that the two can match fail.

## 5. Conclusion

The current new digital technologies are spreading rapidly. The increasing heat of market competition has prompted significant companies to accelerate digital transformation. In the fierce market competition, the digital transformation of HRM becomes the key for companies to enhance their competitive advantages. The development of HRM has a significant positive impact on man-job matching, i.e., career ability development has a positive effect on both required abilities matching and needed supply matching; technical skill training has a positive impact on both required abilities matching and needed supply matching; and performance evaluation feedback has a significant positive effect on both required abilities matching and needed supply matching. In other words, in intelligent manufacturing, technical skills personnel face innovative equipment and techniques facework situations and need to systematically consider design, production, service, and other aspects. Hence, the required technical and professional degree is higher, and the job competency standards also reflect high and high levels. This article combines the theoretical knowledge and practical experience of HRM digitalization. It proposes a general design plan for HRM transformation from digital management based on the design principles of “business orientation, quantitative analysis, and positive feedback.” Based on the design principles of “business orientation, quantitative analysis, and positive feedback,” we conceived a digital transformation plan for HRM based on the three-pillar HRM model, using quantitative indicators, and forming a positive feedback mechanism. Through the continuous optimization of performance indicators, the performance level of HRM can be improved.

## Figures and Tables

**Figure 1:** Human resource management function chart.

**Figure 2:** SCC system job data set.

**Figure 3:** Specific role division and operation management functions.

**Figure 4:** Convolutional neural network model structure.

**Figure 5:** Internet IT jobs salary range.

**Figure 6:** Post data chart.

**Figure 7:** Trend graph of the number of employees.

**Figure 8:** Label prediction results.

**Figure 9:** Effect of different data cut ratio.

## Data Availability

The data used to support the findings of this study are available from the corresponding author upon request.
